# Long noncoding RNA 00460 (LINC00460) promotes glioma progression by negatively regulating miR‐320a

**DOI:** 10.1002/jcb.28232

**Published:** 2019-03-01

**Authors:** Li Feng, Min Rao, Yinan Zhou, Yunxin Zhang, Yonggang Zhu

**Affiliations:** ^1^ Department of Radiotherapy China‐Japan Union Hospital of Jilin University Changchun China; ^2^ Department of Gastroenterology The First Hospital of Jilin University Changchun China; ^3^ Department of the Gastrointestinal Surgery The People's Hospital of Jilin Province Changchun China

**Keywords:** glioma, LINC00460, lncRNA, miR‐320a

## Abstract

**Objective:**

Long noncoding RNA 00460 (LINC00460) has been reported to contribute to tumorigenesis in multiple types of human malignancies. However, the biological role and the underlying molecular mechanism of LINC00460 in glioma remain unclear. The aim of this study was to investigate the clinical value, the biological function, and the potential mechanism of LINC00460 in glioma.

**Methods:**

The expression level of LINC00460 in glioma tissues and cell lines was examined by quantitative real‐time polymerase chain reaction (qRT‐PCR). Cell Counting Kit‐8, flow cemetery, wound healing, and transwell invasion assays were used to explore the effect of LINC00460 on glioma cell proliferation, apoptosis, migration, and invasion. qRT‐PCR and reporter assays were used to further verify the regulatory mechanism of LINC00460 in glioma progression.

**Results:**

LINC00460 expression was upregulated in glioma tissues and cell lines compared with non–tumor brain samples and astrocyte cell line (NHA), respectively. Moreover, increased LINC00460 expression was closely associated with glioma tumor grade. Loss‐of‐function assays revealed that knockdown of LINC00460 significantly inhibited glioma cell proliferation, induced cell apoptosis, and suppressed migration and invasion. The mechanistic assays disclosed that LINC00460 binded to miR‐320a in a sequence‐specific manner and regulated its expression. Moreover, miR‐320 inhibition partially attenuated LINC00460 knockdown‐mediated suppressive effects on glioma cell proliferation, migration, and invasion.

**Conclusion:**

These findings suggested that LINC00460 might function as an oncogenic lncRNA in glioma development and could be explored as a potential therapeutic target for glioma.

## 1 INTRODUCTION

Glioma is the most common type of brain tumor and the most dangerous cancer in humans.^1^ Although great progress has been made in glioma treatment, including surgical resection, radiotherapy, and chemotherapy, the clinical prognosis for patients with glioma remains poor.^2^, ^3^ Thus, exploring the molecular mechanisms engaged in the initiation and development of glioma is crucially important to find the underlying biomarkers and therapeutic targets for this disease.

Long noncoding RNAs (lncRNAs) are a class of noncoding RNAs more than 200 nucleotides in length and have a limited protein‐coding ability.^4^ LncRNAs have been implicated in various biological procession, including cell proliferation, cycle, apoptosis, invasion, and metastasis.^5^ Many lncRNAs have been discovered to be associated with the initiation and development of tumors, suggesting that lncRNAs could serve as diagnostic markers and therapeutic targets for cancer treatment.^6^, ^7^ A number of lncRNAs have been identified to function as oncognenes or tumor suppressors in glioma progression.^8^, ^9^ Thus, exploring novel lncRNAs is an urgent need to understand the mechanism of glioma progression.

Long intergenic noncoding RNA 460 (LINC00460), a newly identified lncRNA, has been reported to be upregulated and to function as an oncogene in several types of cancer, including colorectal cancer,^10^ meningioma,^11^ laryngeal squamous cell carcinoma,^12^ non–small lung cancer,^13^, ^14^ nasopharyngeal carcinoma,^15^ and esophageal squamous cell carcinoma.^16^ However, there is little knowledge about the role of LINC00460 in the progression of glioma. Therefore, our study was aimed at examining the LINC00460 expression level, elucidating the physiological functions of LINC00460, and investigating its molecular mechanism in glioma progression through a series of experiments.

## 2 MATERIALS AND METHODS

### 2.1 Clinical samples and cell lines

A total of 42 pairs of glioma tissues were obtained from volunteer patients with glioma who underwent surgery at the First of Hospital of Jilin University from March 2014 to March 2015. A total of 10 non–tumor brain samples from patients receiving craniocerebral decompression due to traumatic brain injury were collected from our hospital. None of the patients received any antitumor treatment before surgery. All tissues were immediately frozen in liquid nitrogen and stored at −80°C for the subsequent analysis. This study was approved by the Ethics Committee of the First of Hospital of Jilin University, and a written informed consent was received from all patients.

Human astrocyte cell line (NHA) and four glioma cell lines (U87, U251, LN229, and A172) were bought from the American Type Culture Collection (ATCC) and were grown in DMEM (Gibco, CA) containing 10% FBS (Gibco), 2 mM l‐Glutamine, 100 U/mL penicillin/streptomycin at 37°C, and 5% CO_2_.

### 2.2 Quantitative real‐time polymerase chain reaction

Total RNA was extracted from the glioma tissues and normal brain tissues or cultured cells using TRIzol reagent (Invitrogen, Carlsbad, CA) following the manufacturer's instructions. RNA quality and concentration were evaluated by a Nanodrop 2000 (Thermo Fisher Scientific, Wilmington, DE). Total RNA was reverse‐transcribed into cDNA using Prime‐Script RT Reagent Kit (Takara, Dalian, China). Quantitative real‐time polymerase chain reaction (qRT‐PCR) was performed with SYBR Prime Script RT‐PCR kits (Takara) on ABI 7500 Fast Real‐Time PCR system m (Applied Biosystems, Foster City, CA) based on the manufacturer's instructions. The sequences of primers (BGI, Shenzhen, China) used in this study were: LINC00460, 5′‐AATGGTGGTAGGAGGGAGGA‐3′ (forward) and 5′‐CAAGGGGAATGAACACGAGG‐3′ (reverse); GAPDH, 5′‐GGGAGCCAAAAGGGTCA‐3′ (forward), 5′‐GAGTCCTTCCACGATACCAA‐3′(reverse); miR‐320a, 5′‐GGGCTAAAAGCTGGGTTGA‐3′ (forward) and 5′‐CAGTGCGTGTCGTGGAGT‐3′ (reverse). U6 5′‐GCTTCGGCAGCACATATACT‐3′ (forward), and 5′‐GTGCAGGGTCCGAGGTATTC‐3′ (reverse). GAPDH and U6 were used as internal control to detect lncRNA and miRNA, respectively. The 2^−ΔΔ*Ct*^ method was used to detect the gene relative expression level.

### 2.3 Cell transfection

For the silencing of LINC00460, small interfering RNA oligos targeting LINC00460 (si‐LINC00460; 5′‐GUGUCAACAACCUGUUUAAUU‐3′) and negative control scramble (si‐NC, 5′‐UUCUCCGAACGUGUCACGUTT‐3′) were designed and synthesized by GenePharma (Shanghai, China). miR‐320a mimic, miR‐320a inhibitor, and negative control (miR‐NC) were bought from GenePharma.

For transfection, approximately 1000 U87 cells were plated in each well on a 96‐well plate at 37°C in a humidified 5% CO_2_ for 24 hours. Then, 100 nM siRNAs or miRNAs were transfected into U87 cells using Lipofectamine 3000 (Invitrogen) following the manufacturer's instructions. The transfection efficiency was determined 48 hours after transfection by qRT‐PCR.

### 2.4 Cell viability assay

Cell viability was determined using the cell counting kit‐8 (CCK8; Beyotime, Beijing) following the manufacturer's guide. Briefly, transfected cells (2000 cells/well) in each group were plated into 96‐well plates, and cultured for 24 ‐72 hours. The CCK8 regent (~10 μL) was added to each well for 2 hours at 37°C with 5% CO_2_. Afterward, the absorbance was measured at a wavelength of 450 nm using a microplate reader (ELx800; BioTek Instuments, Inc, Winooski, VT).

### 2.5 Cell apoptosis assay

U87 cells were digested with trypsin and harvested 48 hours after transfection. Cell apoptosis was determined using an Annexin V‐FITC Apoptosis Detection Kit (Invitrogen) by FACS Calibur (BD) according to the manufacturer's instructions. The apoptotic rate was calculated using FlowJo Version 6.1 software (TreeStar, Asland, OR).

### 2.6 Wound healing assay

Transfected cells were seed into six plates at a density of 5 × 10^4^ cells/well and grown to 100% confluence. Then, an artificial wound was created using a sterile 100 μL micropipette tip. After being cultured in serum‐free medium for another 24 hours, the cells were photographed under an X71 inverted microscope (Olympus Corporation) at 100× magnification. The migration distance (units) was analyzed using the NIH the ImageJ software (National Institutes of Health, Bethesda, MD).

### 2.7 Transwell invasion assay

Cell invasion was determined using Matrigel transwell invasion assay. Briefly, 48 hours after transfection, 5 × 10^4^ cells in serum‐free DMEM were added into the upper chamber of a BD BioCoat Matrigel Invasion Chamber (BD Biosciences, San Jose, CA) with 8 μm pores and coated with Matrigel matrix (BD Biosciences). Six hundred microliters of a medium containing 20% FBS was seeded into the lower chambers. After being cultured for 48 hours, the noninvaded cells were removed and the invaded cells were fixed in 20% methanol and stained with 0.1% crystal violet. The fixed cells were photographed and counted in five randomly selected fields under an X71 inverted microscope (Olympus Corporation, Tokyo, Japan).

### 2.8 Bioinformatics prediction and luciferase reporter assay

A publicly available algorithm (StarBase v2.0) was used to predict the binding sites between LINC00460 and target miRNAs. The sequence of the LINC00460‐3′‐untranslated region (3′‐UTR) containing a putative binding site of miR‐320a was synthesized and cloned into the pmirGLO dual‐luciferase vector (Promega, Madison, WI). It was referred to as WT‐LINC00460. The putative binding site was mutated using a QuikChange XL Site‐Directed Mutagenesis kit (Agilent Technologies, Santa Clara, CA) and named MT‐LINC00460. Then U87 cells were cotransfected with reporter plasmid WT‐LINC00460 or MT‐LINC00460 and miR‐320a mimics or control mimics (miR‐NC) using Lipofectamine 3000. The luciferase activity was determined at 48 hours after transfection using a Dual‐luciferase Reporter Assay System (Promega) according to the manufacturer's instructions.

### 2.9 Statistical analysis

All results were shown as the mean ± standard deviation (SD) from at least three independent experiments and were analyzed using version 19 SPSS statistical software (SPSS, Chicago, IL). Differences between groups were analyzed using the Student *t* test or one‐way analysis of variance. Spearman's correlation coefficient was used to assess correlations with LINC00460 and miR‐320a. For all statistical analyses, *P* values less than 0.05 were considered statistically significant.

## 3 RESULTS

### 3.1 LINC00460 expression was upregulated in glioma tissues and cell lines

To investigate the role of LINC00460 in glioma progression, we first examined LINC00460 expression in glioma tissues in comparison with the normal brain tissues. qRT‐PCR data showed that that relative expression of LINC00460 was higher in glioma tissues than that in normal brain tissues (Figure 1A). In addition, we also determined the LINC00460 expression level in four glioma cell lines (U87, U251, LN229, and A172) and human astrocyte cell line (NHA). As shown in Figure 1B, the LINC00460 expression was obviously increased in four glioma cell lines, compared with the NHA cells. We also found that the LINC00460 expression was higher in advanced tumor grade (III‐IV) compared with the tumor grade (I‐II) (*P* < 0.01; Figure 1C). These results suggested that LINC00460 might play crucial roles in glioma development.

**Figure 1:** LINC00460 expression was upregulated in glioma tissues and cell lines. A, The expression of LINC00460 was examined in glioma tissues and normal brain tissues by qRT‐PCR. B, The expression of LINC00460 was examined in four glioma cell lines (U87, U251, LN229, and A172) and human astrocyte cell line (NHA). C, The expression of LINC00460 was measured in different tumor grade. *P < 0.05, **P < 0.01. qRT‐PCR, quantitative real‐time polymerase chain reaction

### 3.2 Knockdown of LINC00460 suppressed glioma cell proliferation and induced cell apoptosis

To explore the biological role of LINC00460 in glioma, U87 cells were transfected with si‐LINC00460 and si‐NC. A satisfactory transfection efficiency was obtained at 48 hours after transfection as confirmed by qRT‐PCR (Figure 2A). CCK‐8 assay revealed that knockdown of LINC00460 significantly suppressed cell proliferation in U87 cells (Figure 2B). Flow cemetery assay demonstrated that knockdown of LINC00460 significantly induced cell apoptosis compared with the si‐NC group (Figure 2C).

**Figure 2:** Knockdown of LINC00460 suppressed glioma cell proliferation and induced cell apoptosis. A, The expression of LINC00460 was examined in U87 cells transfected with si‐LINC00460 and si‐NC. B, Cell proliferation was detected in U87 cells transfected with si‐LINC00460 and si‐NC by CCK8 assay. C, Cell apoptosis was detected in U87 cells transfected with si‐LINC00460 and si‐NC by flow cemetery. *P < 0.05, **P < 0.01

### 3.3 Knockdown of LINC00460 suppresses glioma cell migration and invasion

Wound healing and transwell invasion assays were performed to investigate the influence of LINC00460 on the migration and invasion of glioma cells. The results demonstrated that knockdown of LINC00460 significantly suppressed migration and invasion of U87 cells (Figure 3A and 3B).

**Figure 3:** Knockdown of LINC00460 suppressed glioma cell migration and invasion. A, Cell migration was determined in U87 cells transfected with si‐LINC00460 and si‐NC by wound healing assay. B, Cell invasion was determined in U87 cells transfected with si‐LINC00460 and si‐NC by transwell invasion assay. *P < 0.05, **P < 0.01

### 3.4 LINC00460 functioned as a sponge for miR‐320a in glioma

Accumulating evidence indicates that lncRNAs could directly interact with miRNAs by the means of sponging, acting as competing endogenous RNAs (ceRNAs).^17^ To further understand the underlying mechanism by which LINC00460 contributes to promoting glioma progression, starBase v2.0 (http://starbase.sysu.edu.cn/ mirLncRNA.php) software was used to predict the binding sites between LINC00460 and target miRNAs. Among several miRNAs, LINC00460 had a highly predicted binding site with miR‐320a (Figure 4A). Moreover, miR‐320a was reported to be downregulated in glioma tissues and suppressed glioma progression by directly targeting multiple genes.^18^, ^19^ Consistent with the above studies, we also found that miR‐320a expression was significantly downregulated in glioma tissues (Figure 4B; *P* < 0.01). Intriguingly, miR‐320a expression was negatively correlated with LINC00460 expression in glioma tissues (Figure 4C). To further investigate whether LINC00460 could directly interact with miR‐320a, a dual‐luciferase reporter assay was performed. The results indicated that overexpression of miR‐320a could significantly inhibit the reporter activity of WT‐LINC00460 but not MT‐LINC00460 (Figure 4D). Moreover, miR‐320a was increased in U87 cells after the knockdown of LINC00460 expression (Figure 4E), while LINC00460 expression was significantly decreased in U87 cells after transfection with the miR‐320a mimics (Figure 4F). The above results suggested that LINC00460 directly interacted with miR‐320a in glioma cells.

**Figure 4:** LINC00460 functioned as a sponge for miR‐320a in glioma. A, Diagram of putative binding sites and mutant sites between LINC00460 and miR‐320a was shown. B, The expression of miR‐320a was examined in glioma tissues and normal brain tissues by qRT‐PCR. C, Inverse expression correlation between LINC00460 and miR‐320a in glioma tissues (n = 42). D, The luciferase activity was measured in U87 cells cotransfected with a reporter plasmid WT‐LINC00460 or MT‐LINC00460 and miR‐320a or miR‐NC mimic. E, The expression of miR‐320a was examined in U87 cells transfected with si‐LINC00460 and si‐NC by qRT‐PCR. F, The expression of LINC00460 was examined in U87 cells transfected with miR‐320a or miR‐NC mimic. *P < 0.05, **P < 0.01. qRT‐PCR, quantitative real‐time polymerase chain reaction

### 3.5 miR‐320a inhibition partially reversed the effects of LINC00460 knockdown in glioma cells

To obtain direct evidence that the downregulation of miR‐320a was required for the effects of LINC00460, we transfected a miR‐320a inhibitor into LINC00460‐ depleted U87 cells, and the results revealed that miR‐320a was markedly suppressed (Figure 5A).The results of the CCK‐8 assay, flow cytometry, wound healing, and transwell invasion assay showed that the effects mediated by LINC00460 depletion on cell proliferation, apoptosis, migration, and invasion were partly abolished by the introduction of miR‐320a inhibitor in U87 cells (Figure 5B‐E). These results indicated that miR‐320a was involved in the LINC00460‐mediated oncogenic activity.

**Figure 5:** miR‐320a inhibition partially reversed the effects of LINC00460 knockdown in glioma cells. A, Relative expression of miR‐320a was examined by qRT‐PCR in U87 cells transfected with si‐NC, si‐LINC00460, and si‐LINC00460+miR‐320a inhibitor. B‐E, Cell proliferation, apoptosis, migration, and invasion were determined in U87 cells transfected with si‐NC, si‐LINC00460, and si‐LINC00460 + miR‐320a inhibitor. *P < 0.05, **P < 0.01. qRT‐PCR, quantitative real‐time polymerase chain reaction

## 4 DISCUSSION

Recently, lncRNAs have gained wide attention from cancer researcher because they appear to be involved in tumor initiation and development in various types of cancer.^20^, ^21^ A number of lncRNAs were identified to serve as diagnostic markers and therapeutic agents for glioma.^8^, ^9^ Here, we identified a novel lncRNA, LINC00460, which promoted glioma progression. We found that LINC00460 expression was upregulated in glioma tissues and cell lines, and its expression was associated with tumor grade. LINC00460 knockdown suppressed glioma cell proliferation, migration and invasion, and induced cell apoptosis in vitro. Mechanism analysis demonstrated that LINC00460 contributed to glioma cell growth and invasion by sponging miR‐320a.

LINC00460, located at human chromosome 13q33.2, has been reported to be involved in tumor progression in multiple types of cancer.^10^, ^11^, ^12^, ^13^, ^14^, ^15^, ^16^ For example, Lian et al^10^ reported that LINC00460 promoted cell proliferation and inhibited apoptosis by regulating KLF2 and CUL4A expression in colorectal cancer. Xing et al^11^ demonstrated that LINC00460 knockdown significantly suppressed meningioma cell proliferation ability, increased the apoptosis, and decreased the proteins (MMP‐2, MMP‐9, ZEB1) expression by targeting miR‐539. Li et al^14^ found that LINC00460 promoted non–small cell lung cancer cell migration and invasion and epithelial‐mesenchymal transition process by regulating hnRNP K. Kong et al^15^ showed that LINC00460 facilitated nasopharyngeal carcinoma tumorigenesis by sponging miR‐149‐5p to upregulate IL6. However, the biological role of LINC00460 in many cancers, especially in glioma, has not yet been well characterized and needs to be further explored. The present study demonstrated that the expression of LINC00460 was remarkably upregulated in glioma cell lines and tissues, and its expression was positively associated with advanced tumor grade. Loss‐of‐function strategies showed that LINC00460 suppressed glioma progression by inhibiting cell proliferation, migration, and invasion. To the best of our knowledge, this is the first study to demonstrate that LINC00460 may be regarded as an oncogene in glioma.

Accumulating evidence has revealed that lncRNAs could function as miRNA sponges or ceRNA in regulating tumor progression.^22^, ^23^ LINC00460 has been reported to act as a ceRNA for regulating miR‐539 in meningioma^11^ and miR‐149‐5p in nasopharyngeal carcinoma.^15^ To explore the molecular mechanism of LINC00460 in glioma progression, Starbase v.2.0 was used to predict potential miRNAs that directly interacted with LINC00460. Among the target miRNAs, miR‐320a was selected as a potential target based on its biological function in glioma. Previous studies showed that miR‐320a functions as a tumor suppressor in glioma progression by directly targeting multiple genes.^20^, ^21^ Here, we found that miR‐320a expression was significantly downregulated in glioma tissues, which was consistent with previous studies.^20^, ^21^ Intriguingly, miR‐320a expression was negatively correlated with LINC00460 expression in glioma tissues. Moreover, dual‐luciferase reporter assays revealed that overexpression of miR‐320a could significantly inhibit the reporter activity of WT‐LINC00460, but not of MT‐LINC00460. Our results also demonstrated that miR‐320a was increased in U87 cells after the knockdown of LINC00460 expression (Figure 4E), while LINC00460 expression was significantly decreased in U87 cells after transfection with miR‐320a mimics (Figure 4F). Importantly, inhibition of miR‐320a partially reversed the LINC00460 knockdown–mediated inhibitory effect on cell proliferation, apoptosis, migration, and invasion. These findings indicated LINC00460 exhibited important regulatory functions in glioma via sponging miR‐320a.

## 5 CONCLUSION

The current study showed that LINC00460 was upregulated in glioma tissues and cell lines, and its high expression was associated with tumor grade in glioma patients. Furthermore, in vitro experiments indicated that LINC00460 acted as an oncogene in glioma development via sponging miR‐320a. These studies suggested that LINC00460 might be applied as a potential target for glioma therapy.

## CONFLICTS OF INTEREST

The authors declare that they have no conflicts of interest.
